# EPO Receptor Gain-of-Function Causes Hereditary Polycythemia, Alters CD34^+^ Cell Differentiation and Increases Circulating Endothelial Precursors

This article has been retracted.

**DOI:** 10.1371/journal.pone.0012015

**Published:** 2010-08-05

**Authors:** Silverio Perrotta, Valeria Cucciolla, Marcella Ferraro, Luisa Ronzoni, Annunziata Tramontano, Francesca Rossi, Anna Chiara Scudieri, Adriana Borriello, Domenico Roberti, Bruno Nobili, Maria Domenica Cappellini, Adriana Oliva, Giovanni Amendola, Anna Rita Migliaccio, Patrizia Mancuso, Ines Martin-Padura, Francesco Bertolini, Donghoon Yoon, Josef T. Prchal, Fulvio Della Ragione

**Affiliations:** 1 Department of Pediatrics, Second University of Naples, Naples, Italy; 2 Department of Biochemistry and Biophysics “F. Cedrangolo”, Second University of Naples, Naples, Italy; 3 Foundation Ospedale Maggiore Policlinico IRCCS, University of Milan, Milan, Italy; 4 Ematologia-Oncologia Pediatrica, Ospedale di Nocera Inferiore, Nocera Inferiore, Italy; 5 Mount Sinai School of Medicine, New York, New York, United States of America; 6 Laboratory of Hematology-Oncology, European Institute of Oncology, Milan, Italy; 7 Hematology Division, School of Medicine, University of Utah and VAH, Salt Lake City, Utah, United States of America; The University of Hong Kong, Hong Kong

## Abstract

**Background:**

Gain-of-function of erythropoietin receptor (*EPOR*) mutations represent the major cause of primary hereditary polycythemia. EPOR is also found in non-erythroid tissues, although its physiological role is still undefined.

**Methodology/Principal Findings:**

We describe a family with polycythemia due to a heterozygous mutation of the *EPOR* gene that causes a G**→**T change at nucleotide 1251 of exon 8. The novel *EPOR* G1251T mutation results in the replacement of a glutamate residue by a stop codon at amino acid 393. Differently from polycythemia vera, *EPOR* G1251T CD34^+^ cells proliferate and differentiate towards the erythroid phenotype in the presence of minimal amounts of EPO. Moreover, the affected individuals show a 20-fold increase of circulating endothelial precursors. The analysis of erythroid precursor membranes demonstrates a heretofore undescribed accumulation of the truncated EPOR, probably due to the absence of residues involved in the EPO-dependent receptor internalization and degradation. Mutated receptor expression in EPOR-negative cells results in EPOR and Stat5 phosphorylation. Moreover, patient erythroid precursors present an increased activation of EPOR and its effectors, including Stat5 and Erk1/2 pathway.

**Conclusions/Significance:**

Our data provide an unanticipated mechanism for autosomal dominant inherited polycythemia due to a heterozygous *EPOR* mutation and suggest a regulatory role of EPO/EPOR pathway in human circulating endothelial precursors homeostasis.

## Introduction

Erythropoietin (EPO) is a key cytokine, produced mainly in peritubular renal cells but also in the liver, that modulates the growth, survival, and differentiation of erythroid progenitor cells, leading to tight control of red blood cell production. Its receptor (EPOR) is a homodimeric transmembrane protein of 508 amino acids in humans (507 in mice) that belongs to a superfamily of cytokine receptors, which includes receptors for GM-CSF and interleukin-3 and -6 [1]. As with other members, the extracellular ligand binding region of EPOR contains four conserved cysteine residues and a WSXWS motif.

The human *EPOR* gene is located on chromosome 19 and contains eight exons [2 and references therein.] The first five exons encode the extracellular region that embraces the high EPO affinity of A, B, D helix site-1 and the low Epo affinity of A, C helix site-2 interactions, with 7 beta-strand bipartite binding sites in appositioned EPOR dimmers. Exon 6 encodes the membrane spanning domain, while the two intracellular receptor domains are encoded by exons 7 and 8 [2 and references therein].

The receptor does not possess any kinase activity, but its intracellular region binds to JAK2 tyrosine kinase that is essential for EPO signaling. EPOR engagement stimulates JAK2 phosphorylation at Y1007/1008 residues [3]. In turn, activated JAK2 (in concert with other kinases) phosphorylates eight conserved tyrosines in cytoplasmic domain [4]. These phosphotyrosine (PY) sites of EPOR function as docking sites for the binding of molecules containing SH2/SH3 motifs to EPOR. One subset of PY site–recruited factors (PY 402, 430, 432) coordinates negative feedback of EPO signaling. EPO's positive signals are determined by different PY site-recruited factors (PY 344, 426, 461, 465, 480) [4]. It is currently assumed that two boxes at the membrane-proximal region of the EPOR cytoplasmic domain and Y344 are the major positive motifs and that the activation of Stat5 is central for EPOR function [5]. However, since these conclusions have been mainly reached in animal models or in non-erythroid artificial *in vitro* cell systems, these assumptions await confirmation in the physiological human environment.

In the mouse spleen and bone marrow, EPOR engagement regulates erythropoiesis [6], while the EPO importance in brain development and, possibly, in endothelial precursor mobilization has been suggested [7], [8]. Moreover, EPO/EPOR signaling, at least in the mouse, seems to have a protective role in myocardial ischemia/infarction and in pulmonary hypertension [7], [8]. However, the notion that EPOR plays non-erythropoietic function has been recently strongly challenged [9]. It is also to underscore that erythropoiesis is not equivalent in mice and humans. Thus, a transgenic mouse with the mouse *EpoR* gene replaced with human polycythemia-causing *EPOR*, with the truncated deletion in the intracellular region just before tyrosine 410, was polycythemic [10]. Conversely, mice expressing a truncated mouse *EpoR* were not polycythemic [11]. This emphasizes that results obtained in animal models, albeit important for the understanding of gene function, might not be always extrapolated to human physiology and/or human diseases.

EPOR has been reported to be expressed not only in erythroid precursors but also in other cells and organs, including endothelial cells, the brain, and kidneys [8], [12], [13]. These findings have been obtained by immunohistochemical studies, as well as with highly sensitive reverse transcription-polymerase chain reaction [12], [13]. However, strongly concerns have been raised about the specificity of antibodies used to detect EPOR [14], and the presence of EPOR transcripts is not sufficient to demonstrate the occurrence of an active receptor and its downstream pathways. Therefore, the distribution of functional EPOR in human tissues still remains controversial.

The interest in EPOR has recently exploded following reports of the presence of the receptor on cancer cells with detrimental clinical outcome after EPO treatment [15], [16]. Although the role of EPO in cancer progression remains controversial [17], the possible EPOR-dependent proliferation of neoplastic cells highlights the importance of accurate delineation of human EPOR physiology.

A small number of *EPOR* mutations have been described, which are associated with primary familial and congenital polycythemias (PFCPs) [18]–[25]. These patients show, low serum EPO levels, normal haemoglobin oxygen affinities, and erythroid progenitors that exhibit EPO hypersensitivity [26]. Clinically, PFCP patients may present with symptoms ranging from headaches, dizziness, epistaxis, exertional dyspnea to pruritis after bathing [27]. Moreover, thrombotic and hemorrhagic events with premature morbidity and mortality have been reported [28], [29]. Clinical symptoms are effectively relieved by phlebotomy, but the increased risk of cardiovascular morbidity is not ameliorated by maintaining a normal hematocrit [30]. However, detailed cellular and molecular explanations of the mutated EPOR pathophysiology of these patients have not been obtained.

We investigated the *EPOR* gene in a family with dominant polycythemia and found a mutation resulting in a receptor lacking most of the cytoplasmic domain. We demonstrated a marked increase of EPOR protein on the membrane of erythroid progenitors and report its role in deregulating CD34^+^ cells proliferation and differentiation. We also describe a strong increase of circulating endothelial precursors in the affected subjects.

## Results and Discussion

The propositus (**P1,** **Figure 1A**) was referred from a group of 114 patients included in the Italian registry of congenital erythrocytosis/polycythemia. The index patient is a 14-year-old child who, at 7 years of age, was evaluated for persistent headaches and leg muscle cramps. He had an elevated hemoglobin level and hematocrit (21 g% and 66%, respectively), no splenomegaly, and normal blood pressure. White blood cell and platelet counts were normal. The patient's 41-year-old father (P3) presented at 19 years of age with elevated values for hemoglobin and hematocrit (20.1 g% and 64%, respectively) and normal white-cell and platelet counts. He suffered from persistent headaches and had a mild mitral valve insufficiency and a liver steatosis. Both P1 and P3 were regularly phlebotomized with symptomatic relief. The propositus' paternal grandfather was also reported as “polycythemic”. He died at 55 years of age of liver cirrhosis. The hemoglobin level and hematocrit were also elevated in the paternal uncle (P4) and his daughter (P5), but these patients have scarce clinical symptoms and, thus, were not phlebotomized. The serum EPO was <3 mU/mL (normal range, 4 to 32 mU/mL) in all the four polycythemic family members, while hemoglobin oxygen affinities (p50) were normal.

**Figure 1:** EPOR mutation and pedigree of the polycythemic family. **Panel A**. The panel shows nucleotides 1242–1270 (exon 8) of the *EPOR* gene. A heterozygous *G1251* **→** *T* mutation was detected in the propositus P1. The same mutation was verified in all the subjects affected by erythrocytosis (P1, P3, P4, and P5). **Panel B**. Pedigree of the family with dominant familial erythrocytosis is shown. Squares represent males, circles represent females, and Ps represent the subjects that were genotyped. P1, P3, P4, and P5 are the subjects affected by congenital polycythemia.

All patients were screened for defects in the *Von Hippel-Lindau*, *HIF-1alpha*, *HIF-2alpha*, *PHD1-3*, *JAK2*, and *EPOR* genes. No mutations were found in the *Von Hippel-Lindau*, *HIF-1alpha*, *HIF-2alpha*, *PHD1*, *PHD2*, *PHD3*, *and JAK2* genes. However, a heterozygous G**→**T change at nucleotide 1251 in exon 8 of the *EPOR* gene was detected in the index patient (**Figure 1A**). This novel mutation (*EPOR* G1251T) caused the replacement of a glutamic acid residue with a stop codon at amino acid 417, which corresponds to residue 393 of the mature receptor. The *EPOR* G1251T mutation segregated with the polycythemic status, as demonstrated by the *EPOR* analysis of other family members (**Figure 1B**). This genetic change resulted in the synthesis of a truncated receptor lacking the cytosolic tyrosines subjected to phosphorylation, except Y344.

Since our patients had a very low serum EPO level, we investigated the growth and differentiation of erythroid precursors in the absence of exogenously added EPO with normal and polycythemia vera (PV) cells used as controls. PV cells were chosen as their erythroid precursors are EPO hypersensitive.

In a first set of experiments, the proliferation of erythroid precursors was investigated by employing liquid cultures of mononuclear cells as previously reported [31]. The concentration of EPO in these experiments, due to the fetal bovine serum present in the culture medium, was calculated to be 0.4 mU/mL, namely about ten-fold lower that the patient EPO serum and 7–8 thousand-fold lower than the amount used in *in vitro* erythroid precursors cultures (i.e. 3 U/mL). We observed that the peripheral erythroid *EPOR* G1251T precursors grew 2–3 times faster than cells from PV. Thus, the cells from *EPOR* G1251T patients increased about 16-fold after 12 days compared to a 6-fold increase of the PV subjects (**Figure 2A**). Under the same condition, normal erythroid precursors underwent apoptosis. Significant growth rate differences between *EPOR* G1251T and PV patients were evident at all examined time-periods (**Figure 2A**).

**Figure 2:** Phenotypical features of erythroid precursors and CD34^+^cells from the affected patients. **Panel A**. Growth curve of blood erythroid precursors from the the four *EPOR* G1251T subjects, three subjects affected by PV (*JAK2* V617F homozygotes), and three healthy subjects. Erythroid precursors were grown from peripheral mononuclear cells as described (Migliaccio *et al*., 2002) without adding recombinant EPO. The estimated concentration of EPO in the growth medium was about 0.4 mU/mL. Data represent mean ± SEM (n = 3 per cell type), and are representative of 3 experiments. **Panel B**. The graphic reports the percentage of BFU-E cells (evaluated by glycophorin A expression after 14 days growth) in liquid cultures of erythroid precursors from the P1 patient and two PV patients (*JAK2* V617F homozygotes). The cells were cultured in the absence of exogenously added EPO. Data represent mean ± SEM (n = 3 per cell type), and are representative of 2 experiments. **Panel C**. Fluorescent activated cell scanner (FACS) analysis of liquid cultures of peripheral purified CD34^+^ cells grown for 14 days in with minimal EPO. The erythroid precursors were prepared from the P1 subject and from a patient affected by PV associated with a classical *JAK2* mutation (*JAK2* V617F homozygote). GlyA^+^ means glycophorin A positive cells. The results are representative of three independent experiments that gave superimposable results. **Panel D**. FACS analysis of samples shown in panel C. The panel reports the analysis of GlyA levels in cells plotted versus forward scatter. **Panel E**. Peripheral CD34^+^ cells were growth on soft agar in the absence of EPO. The images report the features of colonies from the P1 subject (b, d) or from a subject affected by PV (*JAK2* V617F homozygote) (a, c). The results are representative of four independent experiments that gave superimposable results.

Glycophorin A expressing cells were analyzed after 14 days of proliferation without exogenously added EPO (i.e. at 0.4 mU/mL EPO concentration) as reported in **Figure 2B**. The percentages of *EPOR* G1251T cells and PV patients that expressed the erythroid marker were 53±5% and 13±2%, respectively.

When, the same experiment was performed in the presence of 3 U/mL EPO, no significant difference of erythroid maturation was observed (**Figure 2B** **)**.

A second set of experiments was performed employing CD34^+^ cells prepared from *EPOR* G1251T and PV patients to highlight phenotypic differences of the early hematopoietic precursors from these two forms of erythrocytoses. As shown in **Figures 2C and 2D**, while a significant percentage (51.5±4.1%) of peripheral CD34^+^ cells from P1 (grown for 14 days without exogenously added EPO) expressed glycophorin A, the antigen was not detectable in peripheral CD34^+^ cells from PV patients cultured under the same conditions.

When CD34^+^ cells were cultured on soft agar with minimal EPO (0.4 mU/mL) marked differences in the number and size of colonies were observed after 14 days. As shown in **Figure 2E**, CD34^+^ cells of P1 formed large visibly hemoglobinized colonies while only few small, pale, poorly hemoglobinized colonies were seen in CD34^+^ cells cultures from PV patient (**Figure 2E**). Identical findings were obtained with CD34^+^ cells from P3, P4 and P5 patients (data not reported). We also prepared the DNA from the largest colonies of P1 and examined the status of the *EPOR* gene. No gene conversion was observed and the heterozygosity of *EPOR* G1251T was maintained.

Finally, no difference in the number and size of colonies was observed after 14 days when CD34^+^ cells from control subjects, PV patients or PFCP patients were cultured on soft agar in the presence of 3 U/mL EPO (data not reported).

It has been suggested, although still debated, that EPO/EPOR pathway plays a role in the endothelial cell homeostasis. Thus, we analyzed the number of circulating endothelial precursors (CEPs) of all PCFP patients by flow cytometry. CEPs were identified as CD45^dim^/CD34^+^/VEGFR2^+^ peripheral cells [32]. **Figure 3A** depicts an example of the flow cytometry analysis performed. CEPs were 710±85 cells/mL in the *EPOR*-mutated subjects (**Figure 3B**), which is about 20-fold higher than the CEPs in the age-matched controls. The CEP level of 3 examined PV patients, all having a classical *JAK2* mutation (*JAK2V617F*), were similar to the CEPs content of *EPOR* G1251T subjects **(** **Figure 3B**).

**Figure 3:** Analysis of circulating endothelial precursors from polycythemic patients. **Panel A**. Evaluation of circulating endothelial progenitor cells by cell phenotype. The panel reports the flow cytometric analysis of circulating endothelial precursors from patient P1, **a**) shows the gate made to eliminate platelets and cell debris; **b**) reports the gate for eliminating apoptotic/necrotic cells (7-AAD positive); **c**) shows the gate for enumerating CD34^+^ cells; **d**) indicates the gate made to enumerate CD34^+^ and CD45^neg/dim^ cells; **e**) reports the negative control; and **f**) is the final gate enumerating CD45^neg/dim^, CD34^+^, and VEGFR2^+^ circulating endothelial precursors. The results are representative of several (>10) independent experiments that gave superimposable results. **Panel B**. The panel shows the number of circulating endothelial precursors of normal subjects, the four *EPOR* G1251T patients, and three subjects affected by PV. The results represent the mean (bar, SD) of 4 independent evaluations (each performed in duplicate) of the subjects analyzed. **Panel C**. The panel reports a semiquantitative evaluation of the expression of *EPOR* alleles in erythroid precursors from subjects of the family investigated. Total RNA was prepared from erythroid precursors after 7 days of growth (in the presence of 3 U/mL EPO) and retrotranscribed to cDNA. Then, PCR was performed employing primers specific for the two alleles (ie the wild-type and mutated). The antisense primer of the mutated allele inserted a restriction site for NdeI in the amplified product that allowed distinction between the normal and mutated allele. After the PCR reaction, the mixtures were digested with the Ndel enzyme. The 167 bp product is derived from the wild-type transcript while the 144 bp product is from the mutated EpoR mRNA form. The figure is representative of 5 experiments. **Panel D**. Total RNA (see panel C) was employed to evaluate the content of EPOR alleles (wild type and *EPOR* G1251T) by realtime PCR. Expression was normalized to beta-actin and expressed as a percentage of wild type *EPOR* RNA from a control subject. Each bar represents the mean value ±SD. The figure is representative of 4 experiments. Additional details are reported in the text. **Panel E**. Total RNA were prepared from CD34+ cells (grown 7 days in the presence of EPO) and circulating endothelial precursors. Then, RNA was employed to evaluate the content of EPOR transcript by realtime PCR. Expression was normalized to beta-actin and expressed as a percentage of wild type *EPOR* RNA from CD34+ cells Each bar represents the mean value ±SD. The figure is representative of 5 experiments.

The growth characteristics of the *EPOR* G1251T CD34^+^ cells and the increased levels of peripheral CEPs prompted us to investigate *EPOR* mRNA and protein levels during CD34+ erythroid differentiation *in vitro*.

The expression of both *EPOR* mRNA alleles in erythroid precursors from the four patients was evaluated by semiquantitative PCR (**Figure 3C**) and real-time PCR (**Figure 3D**) after 7 days of cultures in the presence of EPO. Both methods demonstrated that mutant *EPOR* G1251T and wild type *EPOR* alleles were expressed at similar levels and that the total EPOR transcript of the *EPOR* G1251T erythroid precursors corresponds to the EPOR mRNA of erythroid precursors of an healthy subject (**Figure 3D**). This is in accord with results of a previous study on PFCP, although different PCR methods were employed [19].

The realtime PCR approach was also employed to evaluate the expression of the two *EPOR* alleles of primary cultures of CEPs (P1, P3 and P5 patients). The results obtained are identical to those obtained on the eythroid precursors in that both mutant *EPOR* G1251T and wild type *EPOR* alleles were expressed at similar levels (data not shown). It is to underline that CEPs *EPOR* mRNA is easily detectable and that it corresponds to about 10% of *EPOR* mRNA of erythroid precursors, the cells that probably express the major amount of this transcript in the human body (**Figure 3E**). In conclusion, the evaluation of levels of the two *EPOR* mRNA forms indirectly argues that similar amounts of normal and truncated protein receptors may exist in EPOR-expressing cells as reported in previous studies on PCFC.

In order to verify this conclusion, the status of the EPOR protein on the membrane of erythroid precursor cells was investigated. The lack of specific antibodies against the N-terminal region of EPOR has so far hampered direct biochemical analyses of the EPOR peptide. Recently, we have identified and characterized in detail a highly specific antiserum against the extracellular domain of the receptor [33]. To rule out nonspecific crossreactivity by the EPOR antibody and identify the molecular weight of the truncated receptor, we prepared the recombinant wild type and mutated EPOR proteins with an *in vitro* transcription and translation (IVTT) kit. Moreover, we expressed the native and truncated EPOR in a human EPOR–negative cell line, i.e. K562 cells, for further positive controls. As shown in **Figure 4A**, the antiserum against the extracellular domain recognized the wild type EPOR form at 66–67 kDa and the mutated EPOR G1251T form at about 52–53 kDa.

**Figure 4:** Analyses of EPOR protein in erythroid precursors. **Panel A**. Western blot analysis of cellular membranes from the following samples (from the left to right): i) UT-7 cells; ii) untransfected K562 cells (Con); iii) wild-type EPOR transfected K562 cells (WT-EPOR); iv) mutated EPOR transfected K562 cells (MutEPOR); v) *in vitro* transcription/translation (IVTT) control mixture; vi) *in vitro* transcribed and translated wild-type EPOR, and vii) *in vitro* transcribed and translated mutated EPOR. K562 cells were transfected employing pMT21 plasmids encoding wild-type or mutated *EPOR*, while pcDNA3.1 plasmids were employed in the IVTT experiments. UT-7 cells were employed since these cells contain abundant amounts of wild-type EPOR (Della Ragione et al., 2007). Immunoblotting was performed with the antiserum against the N-end of EPOR. The bottom image is the filter, before immunoblotting, and colored with Red Ponceau. The image confirms equal loading of membrane proteins (lanes 2,3 and 4) and IVTT assay mixtures (lanes 6, 7 and 8). The immunoblotting is representative of 4 experiments. **Panel B**. The image on the left reports the immunoblotting analysis of membranes from the following samples (from left to right): I) peripheral CD34^+^ cells from a healthy subject (Con) grown for 7 days with EPO (3 U/mL); ii) peripheral CD34^+^ cells from patient P1 (MutEPOR) growth for 7 days with EPO (3 U/mL); iii) peripheral CD34^+^ cells from a healthy subject (Con) grown for 10 days with EPO (3 U/mL); and iv) peripheral CD34^+^ cells from patient P1 (MutEPOR) grown for 14 days with EPO. The immunoblotting on the right reports cell membranes from K562 cells cotransfected with the wild-type and mutated *EPOR* pMT21 plasmids as standard for the two EPOR forms. The immunoblotting was performed with the antiserum against the N-end of EpoR. The filter was also re-analyzed by antibodies against glucophorin A (immunoblotting at the center). The bottom image was taken to the filter colored with Red Ponceau before immunoblotting. The image confirms the equal loading of membrane proteins. The image is of 3 experiments. **Panel C**. The image on the left reports the immunoblotting analysis of membranes from the following samples (from left to right): i) peripheral CD34^+^ cells from a healthy subject (Con) cultured for 7 days without minimal EPO (0.4 mU/mL); ii) peripheral CD34^+^ cells from patient P1 (MutEPOR) cultured for 7 days without EPO. The immunoblotting at the right reports cell membranes from K562 cells cotransfected with both the wild-type and mutated *EPOR* pMT21 plasmids. The immunoblotting was performed using the antiserum against the N-end of EPOR. The bottom image was taken to the filter colored with Red Ponceau before immunoblotting. The image confirms the equal loading of membrane proteins. The immuniblotting is representative of 3 experiments. **Panel D**. Peripheral CD34^+^ cells from patient P1 were cultured for 7 days with EPO. Then, the cells were added with (or without) 50 µM LLnL for 4 hours. Finally, cell membranes were prepared and analyzed fot EPOR content. The immunoblotting was performed with the antiserum against the N-end of EpoR. The immunoblotting on the left reports cell membranes from K562 cells cotransfected with the wild-type and mutated *EPOR* pMT21 plasmids as standard for the two EPOR forms. **Panel E**. K562 cells were cotransfected with the wild-type and mutated forms of EPOR. Then, K562 cell membranes (Input) were immunoprecipitated with an antiserum directed against the EPOR C-end (IP C-end). Finally, the immunoprecipitated materials (IP) and the supernatant (IP Sup) of the reaction were analyzed with the antiserum directed against the EPOR N-terminus (WB N-end). The blot reports the following samples (from the left): i) IVTT wild-type EPOR; ii) membranes from cotransfected K562 cells (Input); iii) the immunoprecipitated materials (IP); iv) the supernatant of the immunoprecipitation (IP Sup); v) IVTT reaction of mutated EPOR. Note that the asterisk represents the signal due to the heavy chain of antibodies employed in the immunoprecipitation. The signal is immediately up to the band of the truncated receptor. Two different times of exposition are reported (1 minute and 5 minutes) to demonstrate the difference in the ratio of wild type/mutated forms in the input and in the supernatant. The input sample is 1/4 of the supernatant sample. The immunoblotting is representative of 3 experiments.

When the isolated cell membrane fractions from the patient were analyzed, we observed the presence of a strong band at the mutated form and a very faint band at the wild type EPOR. The finding was observed in either CD34^+^ cells grown for 7 and 10 days in the presence of 3 U/mL EPO (**Figure 4B**) or in cells cultured for 7 days in minimal EPO level (0.4 mU/mL) (**Figure 4C**). The analysis of membrane fractions from control erythroid precursors showed a barely detectable band of the wild type protein.

It is to underline that when CD34^+^ cells (both from controls or PCFP subjects) were growth in the presence of EPO they showed similar differentiation as demonstrated by their glycophorin A content (**Figure 4B**). Thus, changes in the truncated EPOR protein levels cannot be ascribed to difference in cellular populations due to variable degree of differentiation.

The unanticipated observation that, even in the presence of high EPO, the lack of a large part of the receptor cytoplasmic domain results in the cell membrane accumulation of mutated EPOR, suggested that the truncated receptor has a slower membrane internalization/degradation and an increased half-life due to the absence of sequences required for receptor internalization and degradation.

In order to confirm this hypothesis, we incubated CD34^+^ cells with a proteasome inhibitor, i.e. LLnL, that has been previously reported to induce membrane EPOR accumulation by hampering the receptor removal [34]. Thus, CD34^+^ cells were cultured for 7 days with EPO and, then, treated for 4 hours with the proteasome inhibitor. As shown in **Fig. 4D**, LLnL treatment causes the increase of wild-type EPOR while scarce change of mutated EPOR level was observed. The finding suggests that the turn-over time of the two forms was considerably different, being the mutated form remarkably more stable.

The observed difference of receptor turn-over is also in accord with data obtained in UT-7 cells, showing EPOR internalization and removal requires ubiquitination of the receptor's C-terminal region [34]. In particular, members of the beta-Trcp family have been shown to participate in the E3 ligase activity responsible for EPOR ubiquitination [35]. Beta-Trcp binds to Ser 462 within the intracellular part of the receptor and contributes to EPOR ubiquitination in the presence of the hormone. The ubiquitination mediated by beta-Trcp is a crucial signal for the C-terminus degradation of EPOR because the point mutation of Ser 462 to Ala blocks EPOR targeting to the proteasome, thereby leading to sustained activation of EPOR(S462A). It is interesting that BaF3 cells, expressing a mutated EPOR unable to bind beta-Trcp, are hypersensitive to EPO, suggesting beta-Trcp-mediated ubiquitination represents a negative modulator of EPO-induced cellular proliferation [35]. This finding is similar to our observation of a strong EPO hypersensitivity of the erythroid precursors possessing the truncated receptor. In addition, the mechanism is in accord with a recent investigation demonstrating that phosphorylated Y429, Y431, and Y479 in the EPOR cytoplasmic domain bind the p85 subunit of PI3 kinase on EPO stimulation and individually are involved in mediating EPO-dependent EPOR internalization [36].

In order to highlight the biochemical consequences of the truncated receptor accumulation, the possibility that the two EPOR isoforms might interact to form a heterodimer was investigated. Thus, the truncated and wild-type EPORs were overexpressed in K562 cells and membrane proteins were incubated with an antiserum directed against the C-terminus. The immunoprecipitated materials were then analyzed with the antiserum directed against the N-terminus and the occurrence of both the native and the truncated proteins was shown. The result obtained demonstrated that the two EPOR isoforms might undergo heterodimerization (**Figure 4E**). However, although the input material contained equal amounts of the two EPOR isoforms and almost all the wild-type receptor was immunoprecipitated, a large excess of the truncated receptor remained in the supernatant (**Figure 4E**). This argues that the wild-type receptor, and thus the truncated EPOR, preferentially form homodimers.

Therefore, we evaluated whether high levels of homodimers of truncated EPOR might result in excessive EPO signaling and/or in an EPOR autoactivation event. To validate these hypotheses, the truncated EPOR was overexpressed in K562 cells and the effect on receptor autophosphorylation and Stat5 phosphorylation was evaluated. As shown in **Figure 5A**, transfection of the truncated receptor induced a number of biochemical changes (i.e. receptor autophosphorylation and STAT5 phosphorylation), even in the absence of exogenously added EPO, suggesting the possibility of autoactivation and/or hypersensitivity of receptor. Since these events occur at level of truncated EPOR similar to those observed in erythroid precursors cells, it is likely that these receptor features might be observed in these cells.

**Figure 5:** EPOR phosphorylation and STAT5 activation in erythroid cells expressing wild type or mutated EPOR. **Panel A**. K562 cells were transfected with the mutated form of EPOR. After 3 days of growth in the absence of exogenously added EPO, K562 cell membranes and total cell extracts were prepared. (On the left) The membranes were analyzed with antibodies against EPOR N-end or against phosphotyrosine. A phosphotyrosine signal occurs only in the transfected cells and at the molecular weight of the mutated EPOR signal. (On the right) Cell extracts was analyzed for STAT5 and phosphoSTAT5 levels by means of specific antibodies. The immunoblotting is representative of 3 experiments. **Panel B**. Purified CD34^+^ cells from a control and P1 subject were grown for 7 days in the presence of EPO. Then, cell membranes were prepared and EPOR content and phosphorylated form were evaluated as in panel A. The immunoblotting is representative of 3 experiments. The data are are representative of 3 experiments. **Panel C**. Purified CD34^+^ cells from a control and P1 subject were grown for 7 days in the presence of EPO. Then, cell extracts were prepared and STAT5 and its phosphorylated form were analyzed as in panel A. The data are are representative of 3 experiments**. Panel D**. Purified CD34^+^ cells from a control and P1 subject were grown for 7 days in minimal EPO (0.4 mU/mL). Then cell extracts were prepared and STAT5 and phosphorylated fprm were analyzed as in panel A. **Note**: We were unable to evidentiate the phosphorylation of mutated EPOR in CD34+ cells grown in minimal EPO. This was probably due to the scarce amount of material available. However, differences in STAT5 activation between the control cells and cells from the patient were evident in panel D.

Then, we investigated the activity of the EPOR-JAK2-STAT5 pathway in CD34^+^ from control and EPOR truncated subjects, grown for 7 days with or without exogenously added EPO. As shown in **Figures 5B and 5C**, in the presence of 3 U/mL EPO, we found a clear increase of receptor and STAT5 phosphorylation. Although we were unable to directly demonstrate the phosphorylation of the truncated EPOR in the absence of the cytokine, we observed, under this condition, the activation of EPOR-dependent pathway by detecting STAT5 phosphorylation in CD34^+^ cells cultured without EPO (**Figure 5D**). The finding was also confirmed by the activation of Erk1/2, which was significantly increased in cells from EPOR truncated subjects, grown for 7 days with EPO (**Figure 6A**). In the presence of minimal amounts EPO, we also found increased Erk1/2 phosphorylation, which suggests greatly augmented activity of the receptor (**Figure 6B**).

**Figure 6:** Transduction pathway status of erythroid precursors. **Panel A**. Cytosolic extracts of CD34^+^ cells, cultured for 7 days in the presence of EPO, were prepared from a healthy subject and patient P1. Then, samples were analyzed for Erk1/2 and phospho Erk1/2 content. **Panel B**. Cytosolic extracts of of CD34^+^ cells, cultured for 7 days in the absence of exogenously added EPO (0.4 mU/mL EPO), were prepared from a healthy subject and patient P1. Then the samples were analyzed for Erk1/2 and phospho Erk1/2 content. **Panel C**. CD34^+^ cells from a healthy subject were grown for up to 14 days in the presence of EPO. Aliquots of cells at days 0, 7, and 14 were removed and cell extracts were prepared. Then, the samples were analyzed for p27^Kip1^ content by immunoblotting. **Panel D**. CD34^+^ cells from a healthy subject and patient P1 were grown for 7 days in the presence of EPO and cellular extracts were prepared. Then, samples were analyzed for p27^Kip1^ content.

An increase of p27^Kip1^ (an inhibitor of cell cycle progression) has been reported during erythroid differentiation of experimental models of erythropoiesis [37]. As reported in **Figure 6C**, we also observed an increase of p27^Kip1^ on different days of CD34^+^ growth in the presence of EPO. Intriguingly, in cells grown for 7 days with EPO, we found an increase of p27^Kip1^ in cells from the *EPOR* G1251T patient compared with cells of the control subject (**Figure 6D**).

In conclusion, in this study, we report that the gain-of-function *EPOR* G1251T mutation results in a marked alteration of growth and differentiation of human CD34+ and in an increase of erythroid progenitors' surface EPOR peptide. Moreover, we observed a profound increase of circulating endothelial precursors in the affected subject. Our data elucidate how the heterozygous *EPOR* gene mutation causes a dominantly inherited polycythemia phenotype and erythroid progenitors' EPO hypersensitivity. We demonstrate for the first time that, although both alleles of the patients were transcribed at similar rates in erythroid precursors and roughly the same as the normal alleles of healthy subjects, the truncated receptor accumulates at very high levels on cellular membranes. This leads to augmented activation of growth and erythroid differentiation of CD34+ observable at EPO levels lower that that necessary to activate CD34+ of PV patients. EPO hypersensitivity might be due to both: i) the remarkable accumulation of truncated EPOR and its autoactivation, and ii) loss of the negative regulatory domain of the *EPOR* G1251T mutant.

The CD34+ cells proliferation and differentiation, observed without exogenous EPO, also demonstrated the EPOR sequence, including Y344, is sufficient to activate the proliferation and differentiation of human erythroid precursor cells. In the same context, the truncated EPOR-dependent activation of Erk2 suggests Erk2 may not require PY480 or phospholipase C-gamma for its activation, as reported by others [2].

The importance of the EPO-EPOR system in erythropoiesis and vasculogenesis was established using mutant mice lacking either the *Epo* or *EpoR* gene [38]. Although these observations are consistent with participation of EPOR in vasculogenesis, the precise contribution of EPOR function in nonhematopoietic tissue remains to be defined, and is the object of intense debate. It has been described that EPO administration can increase the number of CEPs in healthy subjects. It has been postulated that this increase might be due to an EPO-derived stimulation of cytokine production. Our observation that the *EPOR* G1251T patients with activated EPO-EPOR signaling have an increased number of CEPs suggests the CEPs increase may be due to a constitutive EPO receptor activation in this population. An increase in circulating CD34^+^ cells has been described in patients carrying *JAK2* mutations and suffering from myeloproliferative diseases [39]; to our knowledge, this is the first report demonstrating an increased number of endothelial precursors in the circulation of patients with gain-of-function *EPOR* mutations. It remains to be established whether this is due to increased CEP production, increased CEP mobilization, or both mechanisms.

## Materials and Methods

### Mutational analysis and evaluation of *EPOR* mRNA isoforms

Blood samples were obtained from the index patient, his parents and relatives, from healthy controls, and from four patients with PV (with homozygous *JAK2V617F* mutation). All patients gave written informed consent on entering the study, which was approved by the research ethics committee of Second University of Naples, Italy, and the study was conducted according to the Declaration of Helsinki. DNA and RNA were prepared by standard methods. To screen for mutations of the *EPOR* gene, exons 7 and 8 with exon-intron boundaries were amplified by PCR using the following method and primers:

PCR was performed with 30 cycles of denaturation (1 min, 94°C), annealing (1 min, 60°C), and elongation (1 min, 72°C) and the amplified products were analyzed on 2% agarose gels, stained with ethidium bromide. Oligonucleotides used to amplify either exon 7 (362 bp) or 8.1 (301 bp) and exon 8.2 (333 bp) were as follows:

exon 7 forward: 5′-GCCTCTATGACTGGGAGTGG-3′

exon 7 reverse: 5′-GCGCTCTGAGAGGACTTCC-3′

exon 8.1 forward: 5′-GCCTGGGCTTCCCTGCTTCTTGC-3′

exon 8.1 reverse: 5′-TTCGAGGCCAAAGCAGATGAGCA-3′

exon 8.2 forward: 5′-TATCTGGTGCTGGACAAATGGTT-3′

exon 8.2 reverse: 5′-CTGCAGCCTGGTGTCCTAAGAGC-3′

The amplified products were purified and sequenced.

Two independent methods were developed for quantifying the expression of the *EPOR* alleles (ie wild-type and mutated forms). **First**, we designed a primer incorporating a mismatched base, corresponding to the allele with the G1251T mutation, to engineer a restriction site for NdeI in the PCR product. After the PCR reaction, the assay mixture was digested with the NdeI enzyme (Invitrogen, Carlsbad, CA, USA) and only the product from the mutated allele was digested. The mutated allele yielded 2 fragments of 144 bp and 23 bp, and wild type an uncut 167 bp band.

**Second**, a TaqMan assay was performed using the iCycler iQ Real-Time PCR Detection System (Bio-Rad Laboratories, Hercules, CA). We synthesized two probes, one specific for the detection of the wild-type allele, labeled with a FAM dye, and one specific for the mutated allele, labeled with a HEX dye. Each incorporated Locked Nucleic Acids (Sigma-Aldrich, Sigma Chemical Company, St. Louis, MO, USA), a nucleic acid analogue that contains a 2′-O, 4′-C methylene bridge. This bridge restricts the flexibility of the ribofuranose ring and locks the structure into a rigid C3-endo conformation, conferring enhanced hybridization performance and markedly increased stability. The amount of each expressed allele was standardized using wild-type and mutated *EPOR* pcDNA3.1 plasmids. Further details on the methods, as well as on the primers employed, will be provided on request.

### Erythroid precursor cultures

Liquid cultures of erythroid precursors from peripheral blood were prepared by two methodologies. The first utilized peripheral blood mononuclear cells as a source of erythroid progenitors [31], while the second employed the peripheral blood CD34+ cells as a source of progenitors [40]. Soft agar colony assays were performed as described [41]. The colonies were scored after 0, 7, and 14 days and their images captured after 14 days.

### Circulating endothelial cell evaluation

Circulating endothelial precursors were measured by six-color flow cytometry as previously described [32]. Primary cultures of circulating endothelial precursors were prepared as previously described [32].

### Plasmids, cell lines, and protein analysis

The wild-type coding sequence of human EPOR, cloned into the pMT21 expression vector, was kindly provided by Dr. A. D'Andrea. The sequence was mutagenized at the 1251 (G**→**T) position, and the wild-type and mutated *EPOR* sequences were subcloned into the pcDNA3.1 plasmid. These pcDNA3.1 vectors were used to prepare *in vitro* the respective proteins by TNT kits (Promega Italia, Milan, Italy). pMT21 plasmids containing the wild-type and mutated *EPOR* coding sequences were transiently transfected in the human K562 cell line (a negative erythroleukemic EPOR cell line) by standard procedures [33], [42]. The treatments with N-Ac-Leu-Leu-norLeucinal (LLnL) (Merck Biosciences, Darmstadt, Germany) were performed as reported in [34]. Cell membranes were prepared with the Qproteome Cell Compartment Kit (Qiagen, Valencia, CA, USA), while cytosol and nuclei were obtained using NE-PER Nuclear and Cytoplasmic Extraction Reagents (Pierce Biotechnology, Rockford, IL) [33]. Immunoblotting procedures and immunoprecipitation experiments were essentially performed as described [33], [42].

The following antibodies were employed in the immunoblotting and immunoprecipitation experiments. Goat polyclonal antiserum directed against the extracellular domain of EPOR was from Abcam (Abcam, Cambridge, MA); rabbit polyclonal anti C-end of EPOR, Stat5, and phospho-Erk1/2 and mouse monoclonal antibodies anti Erk1/2 and anti-phosphotyrosine (PY20) were from Santa Cruz Biotechnology (Santa Cruz Biotechnology, Santa Cruz, CA); mouse monoclonal antibodies anti phospho-Stat5 were from Upstate Biotechnology (Upstate Biotechnology, Charlottesville, VA); monoclonal antibodies against p27^Kip1^ were from Transduction Laboratories (Transduction Laboratories Lexington, KY).
